This article has been retracted.

# TUSC3 induces autophagy in human non-small cell lung cancer cells through Wnt/β-catenin signaling

**DOI:** 10.18632/oncotarget.17674

**Published:** 2017-05-08

**Authors:** Yun Peng, Jun Cao, Xiao-Yi Yao, Jian-Xin Wang, Mei-Zuo Zhong, Ping-Ping Gan, Jian-Huang Li

**Affiliations:** ^1^ International Medical Center, Xiangya Hospital, Central South University, Changsha 410008, P.R. China; ^2^ Department of Medical Oncology, The Affiliated Cancer Hospital of Xiangya School of Medicine, Central South University, Changsha 410008, P.R. China; ^3^ Department of Oncology, Xiangya Hospital, Central South University, Changsha 410008, P.R. China; ^4^ School of Information Science and Engineering, Central South University, Changsha 410008, P.R. China

**Keywords:** non-small cell lung cancer, A549 cells, tumor suppressor candidate 3, Wnt/β-catenin signaling pathway, autophagy

## Abstract

We investigated the effects of tumor suppressor candidate 3 (*TUSC3*) on autophagy in human non-small cell lung cancer (NSCLC) cells. A total of 118 NSCLC patients (88 males and 30 females) who underwent surgery at our institute were enrolled in the study. Immunohistochemical analysis revealed that TUSC3 protein expression was lower in NSCLC specimens than adjacent normal tissue. Correspondingly, there was greater methylation of *TUSC3* in NSCLC than adjacent normal tissue. After transient transfection of A549 NSCLC cells with constructs designed to up-regulate or down-regulate TUSC3 expression, we analyzed the effects of inhibiting the Wnt pathway (XAV939) and autophagy (chloroquine, CQ) on the behavior of NSCLC cells. We also performed TOP/FOP-Flash reporter assays, MTT assays, Annexin V-FITC/propidium iodide staining, and acridine orange staining to evaluate Wnt/β-catenin signaling, cell proliferation, apoptosis, and autophagy, respectively. Expression of Wnt/β-catenin pathway components and autophagy-related proteins was analyzed using qRT-PCR and Western blotting. We found that TUSC3 inhibited cell proliferation and promoted both apoptosis and autophagy in A549 cells. In addition, TUSC3 increased expression of autophagy-related proteins. It also increased expression of Wnt/β-catenin signaling pathway components and promoted nuclear transfer of β-catenin, resulting in activation of Wnt/β-catenin signaling. TUSC3 thus induces autophagy in human NSCLC cells through activation of the Wnt/β-catenin signaling pathway.

## INTRODUCTION

Non-small cell lung cancer (NSCLC) is the leading cause of cancer-related death in men worldwide [1]. It is estimated that up to 70% of NSCLC patients are diagnosed with advanced-stage disease [2]. Although cytotoxic chemotherapy is beneficial for patients with advanced NSCLC, the response rate is only 20%−35% and the median survival is 10−12 months [3]. Differences in the clinical presentation of NSCLC patients can be attributed to the diverse molecular mechanisms that drive malignant transformation and dissemination of the primary tumor. Although there have been advances in NSCLC treatment, the prognosis of NSCLC patients is still poor [4]. Autophagy contributes to a variety of pathological processes including tumorigenesis. Inhibition of autophagy is an attractive therapeutic strategy because it can weaken the ability of tumor cells to clear protein aggregates or damaged organelles [5]. A better understanding of the mechanisms of cell death could lead to the development of more effective therapeutics for NSCLC.

Tumor suppressor candidate 3 (*TUSC3*), located on chromosomal band 8p22, was initially characterized as a tumor suppressor gene. It also has vital roles in embryogenesis and cellular metabolism [6]. *TUSC3* is frequently inactivated or lost in various human cancers including prostate, pancreatic, breast, and ovarian cancer [6–9]. Interestingly, silencing of *TUSC3* in ovarian and prostate cancer cells promotes cell proliferation, invasion, and migration [7]. However, up-regulation of *TUSC3* expression has been observed in patients with papillary thyroid carcinoma suggesting it acts as an oncogene [10]. Thus, the role of TUSC3 in carcinogenesis has not been established. A previous study demonstrated that the Wnt/β-catenin signaling pathway can promote autophagy in prostate cancer cells. This pathway is often regulated by tumor suppressor genes in lung and other types of cancer [11, 12]. We therefore investigated whether TUSC3 expression was associated with NSCLC patient prognosis, and whether TUSC3 could promote autophagy in NSCLC cells by regulating Wnt/β-catenin signaling. Our data indicate that TUSC3 is a promising prognostic marker in NSCLC.

## RESULTS

### TUSC3 protein expression is reduced in NSCLC compared to adjacent normal tissue

TUSC3 protein expression was predominantly observed in the cytoplasm. The positive TUSC3 expression rate in NSCLC tissue (32.20%) was lower than in adjacent normal tissue (59.32%) (*P* < 0.05) (Figure 1). The positive TUSC3 expression rate in patients with poorly/undifferentiated tumors (17.24%) was significantly lower than in patients with moderately/highly differentiated tumors (37.08%). Additionally, the positive TUSC3 expression rate in stage III/IV NSCLC patients (14.06%) was lower than in stage I/II patients (53.70%) (both *P* < 0.05). TUSC3 expression was not associated with patients age or gender (both *P* > 0.05) (Table 1).

**Figure 1:** Comparison of TUSC3 protein expression in NSCLC and adjacent normal tissue **(A)** TUSC3 expression in adjacent normal tissue (× 200); **(B)** TUSC3 expression in NSCLC tissue (× 200); **(C)** histograms showing the positive rate of TUSC3 protein expression in NSCLC and adjacent normal tissue; *, *P* < 0.05 compared to adjacent normal tissue; NSCLC, non-small cell lung cancer; TUSC3, tumor suppressor candidate 3.

**Table 1:** The association between TUSC3 protein expression and the clinicopathological features of NSCLC patients

Clinicopathological features	Number of cases	TUSC3		Positive expression rate (%)	*P*
		−	+		
Age (years)					
< 58	58	37	21	36.21	0.360
≥ 58	60	43	17	28.33	
Gender					
Male	88	60	28	31.82	0.878
Female	30	20	10	33.33	
Differentiation					
Moderately/highly differentiated	89	56	33	37.08	0.047
Poorly/undifferentiated	29	24	5	17.24	
TNM stage					
Stage I/II	54	25	29	53.7	< 0.001
Stage III/IV	64	55	9	14.06	

TUSC3: tumor suppressor candidate 3; NSCLC: non-small cell lung cancer; TNM: tumor node metastasis.

### TUSC3 methylation in NSCLC and adjacent normal tissue

The rate of TUSC3 methylation was significantly higher in NSCLC compared to adjacent normal tissue (P < 0.05; Figure 2).

**Figure 2:** Comparison of the TUSC3 methylation rate between NSCLC and adjacent normal tissue; *, P < 0.05 compared to adjacent normal tissue

### TUSC3 expression in six different human NSCLC cell lines

We next examined TUSC3 mRNA and protein expression in six different NSCLC cell lines using qRT-PCR and Western blotting. Varying levels of TUSC3 mRNA and protein were observed in A549, GLC-82, H322, H460, SPC-A1, and HBE human NSCLC cells. A549 cells had the highest TUSC3 expression at both the mRNA and protein levels (Figure 3). Therefore, the A549 cell line was selected for the following experiments.

**Figure 3:** TUSC3 mRNA and protein expression in human NSCLC cell lines (A549, GLC-82, H322, H460, SPC-A1, and HBE) **(A)** Relative TUSC3 mRNA expression in the six NSCLC cell lines analyzed by qRT-PCR; **(B)** Western blot analysis of TUSC3 protein expression in the six NSCLC cell lines; NSCLC, non-small cell lung cancer; TUSC3, tumor suppressor candidate 3; qRT-PCR, quantitative real-time polymerase chain reaction.

### Transfection efficiency of human NSCLC A549 cells

Eight hours after transfection, we observed GFP fluorescence in the vector control, TUSC3, TUSC3 siRNA, and β-catenin siRNA groups. The transfection efficiency in these groups was > 98% (Figure 4A). We analyzed TUSC3 mRNA expression in the five groups by qRT-PCR. As expected, TUSC3 mRNA expression was significantly up-regulated in the TUSC3 group compared to the blank group, and significantly down-regulated in the TUSC3 siRNA group (all *P* < 0.05). There were no significant differences in TUSC3 mRNA expression between the blank, vector control, and β-catenin siRNA groups (all *P* > 0.05) (Figure 4B).

**Figure 4:** Transfection efficiency of human NSCLC A549 cells in the blank, vector control, TUSC3, TUSC3 siRNA, and β-catenin siRNA groups **(A)** GFP expression in A549 cells visualized by fluorescence microscopy; **(B)** analysis of TUSC3 mRNA expression in the five groups by qRT-PCR following transfection; NSCLC, non-small cell lung cancer; TUSC3, tumor suppressor candidate 3; qRT-PCR, quantitative real-time polymerase chain reaction.

### Wnt/β-catenin signaling pathway activity

Luciferase activity was significantly increased in the TUSC3 group compared to the blank group, while activity in the TUSC3 siRNA, β-catenin siRNA, and XAV939 groups was significantly decreased (all *P* < 0.05; Figure 5). No significant differences in luciferase activity were observed between the blank, vector control, and TUSC3 + XAV939 groups (all *P* > 0.05).

**Figure 5:** Analysis of Wnt/β-catenin signaling pathway activity in the blank, vector control, TUSC3, TUSC3 siRNA, β-catenin siRNA, XAV939, and TUSC3 + XAV939 groups using TOP/FOP-Flash reporter assays *, *P* < 0.05 compared to the blank group; TUSC3, tumor suppressor candidate 3.

### TUSC3 inhibits the proliferation of A549 NSCLC cells

MTT assays and proliferation curves revealed a low rate proliferation in the TUSC3 group compared to the blank and vector control groups. Beginning on the third day, the OD values in the TUSC3 group were lower than in the blank and vector control groups (all *P* < 0.05). However, there were no significant differences in the OD values between the blank, vector control, and TUSC3 + XAV939 groups (all *P* > 0.05) (Figure 6). These results demonstrated that *TUSC3* could inhibit the growth of A549 NSCLC cells.

**Figure 6:** MTT assay growth curves for A549 cells in the blank, vector control, TUSC3, TUSC3 siRNA, and TUSC3 + XAV939 groups A reduction in the growth of TUSC3 over-expressing ells was observed 3 days post-transfection. *, *P* < 0.05 compared to the blank and vector control groups; TUSC3, tumor suppressor candidate 3.

### TUSC3 promotes apoptosis in NSCLC A549 cells

We analyzed the rates of apoptosis and necrosis in transfected cells using Annexin V-FITC/PI staining (Figure 7). Interestingly, the early apoptosis rates of A549 cells (the Annexin-positive rate) in the blank, vector control, TUSC3, TUSC3 siRNA, and TUSC3 + XAV939 groups were 1.70 ± 0.42%, 1.82 ± 0.47%, 2.86 ± 0.77%, 1.78 ± 0.39%, and 2.24 ± 1.82%, respectively. The rates of cell necrosis (the PI-positive rate) were 5.25 ± 0.44%, 5.63 ± 0.61%, 18.73 ± 1.84%, 2.89 ± 0.76%, and 5.97 ± 0.89%, respectively. There were no significant differences in the early apoptosis or cell necrosis rates between the blank, vector control, and TUSC3 + XAV939 groups (all *P* > 0.05). The early apoptosis rate remained low in the five groups and no statistically significant differences were observed between groups (all *P* > 0.05). However, the percentage of necrotic cells was significantly higher in the TUSC3 group than in the blank, vector control, TUSC3 siRNA, and TUSC3 + XAV939 groups (all *P* < 0.05). In addition, the rate of apoptosis was significantly lower in the TUSC3 siRNA group than in the blank group (both *P* < 0.05). We analyzed the expression of apoptosis-related proteins and observed elevated expression of Caspase 3 and Bcl2-associated X (Bax)/B-cell lymphoma-2 (Bcl-2) proteins in the TUSC3 group compared to the blank group. In contrast, the levels of these proteins were significantly reduced in the TUSC3 siRNA group (all *P* < 0.05).

**Figure 7:** Analysis of apoptosis in the blank, vector control, TUSC3, TUSC3 siRNA, and TUSC3 + XAV939 groups measured by Annexin V-FITC/PI staining and Western blotting **(A)** Flow cytometry analysis of the rate of apoptosis in A549 cells; **(B)** rates of apoptosis and necrosis in A549 cells; **(C)** expressions of apoptosis-related proteins in A549 cells; **(D)** protein bands of apoptosis-related proteins in A549 cells; *, *P* < 0.05 compared to the blank and vector control groups; TUSC3, tumor suppressor candidate 3; PI, propidium iodide.

### TUSC3 promotes autophagy in A549 NSCLC cells

We next performed acridine orange staining to determine whether TUSC3 could promote autophagy in A549 NSCLC cells. Masses consisting of orange acidophilic granules were observed in the cytoplasm of A549 cells in the TUSC3 group. These structures were likely autophagosomes (Figure 8). The ratios of acidophilic granules in the blank, vector control, TUSC3, TUSC3 + XAV939, TUSC3 siRNA, and TUSC3 + CQ groups were 2.24 ± 0.97%, 2.39 ± 0.83%, 9.36 ± 1.08%, 3.28 ± 1.02%, 1.28 ± 0.42%, and 2.86 ± 0.98%, respectively. The ratio of autophagy was higher in the TUSC3 than in the blank and vector control groups (*P* < 0.05 for both), and there were no significant differences in the autophagy ratios between the blank, vector control, TUSC3 + XAV939, and TUSC3 + CQ groups (all *P* > 0.05).

**Figure 8:** Cell autophagy in the blank, vector control, TUSC3, TUSC3 + XAV939, TUSC3 siRNA, and TUSC3 + CQ groups detected by acridine orange staining **(A)** Acridine orange staining of A549 cells in the six groups; **(B)** comparison of the cell autophagy ratio among the six groups; *, *P* < 0.05 compared to the blank and vector control groups; TUSC3, tumor suppressor candidate 3; CQ, inhibitor chloroquine.

### TUSC3 promotes expression of Wnt/β-catenin signaling pathway and autophagy-related proteins in A549 NSCLC cells

Next, we evaluated the relative expression of Wnt/β-catenin signaling pathway components and autophagy-related proteins in A549 NSCLC cells using qRT-PCR (Figure 9A). No significant differences in β-catenin, GSK-3β, LC3, or Beclin1 mRNA expression were observed between the blank and vector control groups (all *P* > 0.05). β-catenin, LC3, and Beclin1 mRNA expression was significantly increased in the TUSC3 compared to the blank and vector control groups, while GSK-3β mRNA expression was significantly decreased (all *P* < 0.05). We also observed down-regulation of β-catenin, LC3, and Beclin1 mRNA expression in the TUSC3 siRNA group but up-regulation of GSK-3β mRNA expression (all *P* < 0.05). The mRNA expression of β-catenin, LC3, and Beclin1 in the TUSC3 + XAV939 and TUSC3 + CQ groups was significantly decreased compared to the TUSC3 group, while the mRNA expression of GSK-3β was significantly increased (all *P* < 0.05). However, there were no significant differences in β-catenin, LC3, GSK-3β, and Beclin1 mRNA expression between the TUSC3 + XAV939, TUSC3 + CQ, blank, and vector control groups (all *P* > 0.05). Western blotting (Figure 9B) indicated that there were no significant differences in β-catenin, p-β-catenin, p-GSK-3β^Ser9^, LC3 II/LC I, or GSK-3β protein expression between the blank and vector control groups (all *P* > 0.05). No significant differences in β-catenin and GSK-3β protein expression were observed in the TUSC3 group compared to the blank and vector control groups. However, p-β-catenin, LC3 II/LC I, and Beclin1 protein expression were significantly elevated and p-GSK-3β^Ser9^ expression was significantly reduced (all *P* < 0.05). No significant differences in β-catenin and Beclin1 protein expression were observed in the TUSC3 siRNA group. However, we did observe decreased p-β-catenin, LC3 II/LC I, and GSK-3β expression, and increased p-GSK-3β^Ser9^ expression (all *P* < 0.05). The TUSC3 + XAV939 and TUSC3 + CQ groups had lower p-β-catenin, LC3 II/LC I, and Beclin1 expression, and higher p-GSK-3β^Ser9^ expression compared to the TUSC3 group (all *P* < 0.05). However, there were no significant differences between the TUSC3 + XAV939, TUSC3 + CQ, blank, and vector control groups (all *P* > 0.05).

**Figure 9:** The mRNA and protein expression of Wnt/β-catenin signaling pathway components and autophagy-related proteins in the blank, vector control, TUSC3, TUSC3 + XAV939, TUSC3 siRNA, and TUSC3 + CQ groups **(A)** The mRNA expression of Wnt/β-catenin signaling pathway components and autophagy-related proteins detected by qRT-PCR; **(B)** Western blot analysis of the expression of Wnt/β-catenin signaling pathway and autophagy-related proteins; *, *P* < 0.05 compared to the blank and vector control groups; TUSC3, tumor suppressor candidate 3; CQ, inhibitor chloroquine; qRT-PCR, quantitative real-time PCR.

### TUSC3 promotes nuclear transfer of β-catenin in A549 NSCLC cells

The expression and localization of β-catenin was analyzed by immunofluorescence. β-catenin in A549 cells was mainly expressed in the cytoplasm and to a much lesser extent in cell nuclei in the blank, vector control, and TUSC3 siRNA groups (Figure 10). In contrast, β-catenin accumulated in the nuclei of A549 cells in the TUSC3 group, which significantly differed compared to the blank and vector control groups (all *P* < 0.05). In the TUSC3 + XAV939 group, β-catenin was localized in the cytoplasm, and no obvious expression was observed in cell nuclei. Additionally, no significant differences were observed between the TUSC3 + XAV939, blank, and vector control groups (all *P* > 0.05).

**Figure 10:** Immunofluorescence analysis ofβ-catenin expression in the blank, vector control, TUSC3, TUSC3 + XAV939, and TUSC3 siRNA groups **(A)** Fluorescence images showing expression of β-catenin in the five groups; **(B)** histograms showing expression of β-catenin in the five groups; *, *P* < 0.05 compared to the blank and vector control groups; TUSC3, tumor suppressor candidate 3.

## DISCUSSION

The majority of patients with NSCLC present with locally advanced or metastatic disease [13]. In this study, we investigated the molecular mechanisms underlying NSCLC development and progression. Our data indicate that TUSC3 promotes autophagy in NSCLC cells though activation of the Wnt/β-catenin signaling pathway.

Statistical analyses showed that TUSC3 expression was significantly lower in NSCLC compared to adjacent normal tissue, suggesting that loss of TUSC3 expression may promote NSCLC development and progression. TUSC3 was initially thought to function as a tumor suppressor based on a systematic cloning analysis of the 8p22 chromosomal region [14]. Down-regulation of TUSC3 expression has been observed in various cancers including prostate, breast, oral, and ovarian cancer [9]. Loss of TUSC3 expression was shown to result from homozygous deletion of the 8p22 chromosomal region in prostate cancer and promoter hypermethylation in ovarian cancer [15]. Our data indicate that TUSC3 expression is positively associated with TNM stage and tumor differentiation in NSCLC. Consistent with these results, Horak et al. observed reduced TUSC3 protein expression in 13.3% of tissue samples from patients with prostate cancer. However, follow-up studies failed to detect a relationship between TUSC3 and progression-free or overall survival in prostate cancer patients [7]. Down-regulation of TUSC3 expression has also been observed in higher-grade ovarian cancer tissue [14].

We found that the rate of apoptosis and expression of apoptosis-related proteins (Caspase 3 and Bax/Bcl-2) were lower in the TUSC3 siRNA group compared to the blank control group. However, the expression of these proteins was higher in the TUSC3 group, implying that down-regulation of TUSC3 promotes cell proliferation and resistance to apoptosis in NSCLC. TUSC3 is a homologue of the yeast protein Ost3p, which is a subunit of the oligosaccharyl transferase complex, an integral membrane protein complex that catalyzes the N-linked glycosylation of proteins in the endoplasmic reticulum [16, 17]. Several studies have demonstrated that TUSC3 can impact cell proliferation and apoptosis through induction of endoplasmic reticulum stress (owing to the structural similarity between TUSC3 and the yeast Ost3p proteins, which could affect N-linked glycosylation) [18, 19]. N-linked glycosylation is a ubiquitous posttranslational modification of eukaryotic proteins, and alterations in glycosylation have been associated with carcinogenic processes such as invasion and metastasis. Therefore, it is possible that TUSC3 impacts cancer pathogenesis via glycosylation [20, 21]. Fan et al. reported that loss of TUSC3 expression promoted cell proliferation, invasion, and metastasis in pancreatic cancer, and that the inhibitory role of TUSC3 in pancreatic cancer may be associated with enhanced NF-κB activity [6]. Furthermore, Vaňhara et al. demonstrated that silencing of TUSC3 enhanced cell proliferation and migration *in vitro* in ovarian cancer [21]. Importantly, Li et al. found that silencing of TUSC3 suppressed A549 cell growth and proliferation and promoted apoptosis after radiotherapy under hypoxic conditions. These results are consistent with our data [22].

We determined that the autophagy ratio, as well as Beclin, p-β-catenin, and LC3 II/LC I expression were increased in the TUSC3 group, but decreased in the TUSC3 siRNA group compared to the blank and vector control groups, suggesting that overexpression of TUSC3 accelerates autophagy in NSCLC cells through activation of the Wnt/β-catenin signaling pathway. Wnt/β-catenin signaling plays a critical role during embryogenesis as well as carcinogenesis [23]. For example, activation of Wnt/β-catenin signaling can promote the proliferation of embryonic, intestinal, hematopoietic, skin, and neural stem cells and induce the self-renewal and differentiation of stem-like cells [24–27]. In A549 lung adenocarcinoma cells, loss of *TUSC3* gene expression could inhibit autophagy by elevating the level of the nucleoporin p62, which directly associates with GABARAP family members and LC3 to regulate autophagy [22]. These findings are consistent with our data. However, the mechanism by which TUSC3 activates Wnt/β-catenin signaling to promote autophagy in NSCLC is not yet known.

We have shown that overexpression of TUSC3 may promote activation of the Wnt/β-catenin signaling pathway, which contributes to NSCLC development and progression. Our data provide new insights into the role of TUSC3 in NSCLC and indicate that TUSC3 may be a potential therapeutic target. These finding must be confirmed by further studies with larger sample sizes and complementary experimental techniques.

## MATERIALS AND METHODS

### Ethics statement

The Ethics Committee of Xiangya Hospital, Central South University, approved this study. Written informed consent was obtained from all study subjects and/or their legal guardians.

### Study subjects

Tissue specimens were collected from 118 NSCLC patients who underwent surgical treatment at Xiangya Hospital, Central South University, between August 2014 and October 2015. Pathological analysis confirmed the NSCLC diagnosis. Of the 118 NSCLC patients, 58 were < 58 years of age and 60 were ≥ 58 years of age. There were 88 male and 30 female patients, with a mean age of 56.5 ± 12.3 years. There were 29 patients with poorly/undifferentiated tumors, and 89 cases with moderately/high differentiated tumors. According to the TNM staging system [28], 18 patients had stage I, 36 had stage II, 25 had stage III, and 39 had stage IV NSCLC. Lymph node metastasis was observed in 70 patients. The inclusion criteria were the following: (1) recurrent and metastatic NSCLC following conventional therapy, which was diagnosed by a pathological and/or cytological examination; (2) Eastern Cooperative Oncology Group (ECOG) performance status score of 0−2 and expected survival time ≥ 3 months [29]; (3) no major organ dysfunction; (4) no treatment with other chemotherapeutic drugs 4 weeks prior to surgery; and (5) no history of an allergic reaction to a biological agent. The exclusion criteria were: (1) patients who were pregnant, lactating, or childless; (2) uncontrolled primary brain tumors or metastatic tumors of the central nervous system; (3) unhealed purulent or chronically infected wound; (4) liver and kidney dysfunction, or other cardio-cerebrovascular diseases such as coronary heart disease, angina pectoris, myocardial infarction, arrhythmia, cerebral infarction, and cerebral hemorrhage; and (5) history of a mental illness that is not easily controlled. Patients with chronic obstructive pulmonary disease were also excluded from the study. No patients received chemotherapy or radiotherapy prior to surgery. Paired NSCLC and normal mucosal tissue samples (5 cm away from the edge of the NSCLC tissue) were frozen in liquid nitrogen and stored at −70°C. Additional tissue specimens were formalin-fixed (10% formalin) and paraffin-embedded for immunohistochemical analysis.

### Immunohistochemistry

TUSC3 protein expression was analyzed by immunohistochemistry using the PV-9000 two-step method. Serial formalin-fixed, paraffin-embedded tumor microarray sections (4 μm thick) were deparaffinized and rehydrated in a graded series of alcohol. Antigen retrieval was performed using the microwave method. Endogenous peroxidase activity was blocked using 3% hydrogen peroxide. The sections were then incubated with a monoclonal mouse anti-human TUSC3 primary antibody diluted 1: 500 (Cell Signaling Technology, Beverly, MA, USA) at 4°C overnight, followed by a 20 min incubation with polymeric adjuvants at room temperature. Following the incubation, the sections were incubated with an HRP-conjugated monoclonal goat anti-mouse secondary antibody (Abcam, Cambridge, UK) for 30 min at room temperature. Finally, the sections were stained with diaminobenzidine (DAB) (Sigma-Aldrich, St. Louis MO, USA), counterstained with hematoxylin, and mounted on slides for imaging. PBS was substituted for the primary antibody as a negative control, and positive TUSC3 protein expression was indicated by brown or tan cytoplasmic staining. We randomly selected four high-power fields (× 400) in each section containing approximately 200 cells in each field of view. The percentage of positive cells was recorded as follows: (positive tumor cells/total tumor cells) > 10% was considered positive (+) and (positive tumor cells/total tumor cells) ≤ 10% was considered negative (−) [30]. The immunohistochemical results were evaluated by two individuals using the double-blind method.

### Analysis of *TUSC3* methylation

We analyzed *TUSC3* methylation in DNA extracted from NSCLC and adjacent normal tissue. The methylation-sensitive primers were as follows: upstream: 5′-GGTCGGGTAGGCGTGGTGCG-3′; and downstream: 5′-CCGCCCCGCTTACCTACG ACGT-3′, and the non-methylation-sensitive primers were the following: upstream: 5′-GAGGTTGGTTGGGTAGGTGTGGTGG-3′; and downstream: 5′-CACAACCACCACCCCACTTACCTACAACAT-3′. The PCR conditions were as follows: pre-denaturation at 95°C for 5 min followed by 40 cycles of denaturation at 95°C for 1 min, annealing at 60°C for 50 s, and extension at 72°C for 50 s, and a final extension at 72°C for 10 min. Agarose was dissolved in TBE buffer to a final concentration of 2%, heated in the microwave and then cooled to 60°C. Ethidium bromide was added to a final concentration of 0.5 mg/mL. We loaded 8 μL of each amplification product into the gel and ran the gel for 25 min at 100 V. PCR products were imaged under ultraviolet light. The presence of methylated DNA was indicated by the presence of PCR products specific to the methylation-sensitive primers. If PCR products were only observed with the methylation-sensitive primers, the DNA was considered completely methylated. If a mixture of PCR products was observed with both sets of primers, the DNA was considered partially methylated. If PCR products were only observed with the non-methylation-sensitive primers, the DNA was considered non-methylated. Both complete and partial methylation were considered methylation-positive. Double-distilled water was used in place of the primers as a negative control.

### Cell culture

Human NSCLC cell lines (A549, GLC-82, H322, H460, SPC-A1 and HBE) were obtained from the Cell Bank at the Chinese Academy of Sciences (Shanghai, China) and maintained in RPMI-1640 medium (Gibco, Grand Island, NY, USA) supplemented with 10% fetal bovine serum (FBS) (HyClone, Logan, Utah, USA) at 37°C in a 5% CO_2_ environment with 95% humidity (Thermo Scientific Series 8000 incubator; Thermo Scientific, Waltham, MA, USA). The cultured cells displayed monolayer growth and the attachment rate should reach 90% during passage. After aspiration of culture medium, the cells were rinsed twice with PBS and digested by 0.25% trypsin (Gibco, Grand Island, NY, USA). When the intercellular space increased, the trypsin was aspirated. Subsequently, the single cell suspension was prepared by RPMI-1640 culture medium containing 10% FBS, followed by routine passage.

### Plasmid construction

The PLKO.1-sP6-GFP plasmid was purchased from Sigma-Aldrich Chemical Company (St Louis, MO, USA), and the Sclerostin siRNA was synthesized by Shanghai GenePharma Co., Ltd. (Shanghai, China). Oligonucleotides were diluted to 200 μmol/L, denatured at 95°C for 5 min, and annealed at 70°C for 10 min. The annealed mixture was then diluted to 10 nmol/L. Double-stranded oligomers were inserted into the PLKO.1-sP6-GFP vector using the AgeI and EcoRI restriction sites. The reactions (10 μL of total volume: 5 μL of 2X Ligase Buffer, 2 μL of double-stranded DNA oligomers, 1 μL of PLKO.1-sP6-GFP, 1 μL of 1 U/μL T4 ligase, and 1 μL of sterile water) were incubated at 22°C for 3 h. The ligated TUSC3 overexpression and TUSC3 siRNA plasmids were transformed into DH5α cells and cultured overnight at 37°C.

### Transfection of human NSCLC cell lines

A549 NSCLC cells were randomly divided into the following groups: (1) blank (untransfected); (2) vector control (transfected with empty vector); (3) TUSC3 (overexpression vector; upstream primer: 5′-CCTCAGCGGCAGTGTTCTG-3′; downstream primer: 5′-CCTCATCATAGTCCACCATACTGAA-3′) (Sangon Biotech Co., Ltd., Shanghai, China); (4) TUSC3 siRNA (purchased from Sigma-Aldrich); and (5) β-catenin siRNA (upstream primer: 5′-AGCUGAUAUUGAUGGACAG dTdT; downstream primer: 5′-CUGUCCAUCAAUAUCAGCU dTdT-3′). Approximately 6-8 h post-transfection, the culture medium was exchanged. The medium was replaced again after 24 h post-transfection. After 48 h post-transfection, the green fluorescent protein (GFP) expressions were observed by fluorescence microscopy. A fraction of the cells in the blank and TUSC3 groups were collected and treated with XAV939, an inhibitor of the Wnt/β-catenin signaling pathway, at a concentration of 100 nM to generate the XAV939 and the TUSC3 + XAV939 groups, respectively. Sterile double-distilled water was used to dissolve the autophagy inhibitor, chloroquine (CQ, Sigma-Aldrich), to a final concentration of 50 μM [31]. The TUSC3 + CQ group was generated by treating a fraction of the cells from the TUSC3 group with CQ for 24 h.

### TOP/FOP-Flash reporter assays

One day prior to transfection, the cells in the blank, vector control, TUSC3, TUSC3 siRNA, β-catenin siRNA, XAV939, and TUSC3 + XAV939 groups were inoculated into 24-well plates at 5 × 10^4^ cells/well The pRL-sv40 plasmid (internal control) purchased from Promega Corp. (Madison, Wisconsin, USA) was transfected into cells in the seven groups along with the TOP/FOP-Flash reporter plasmid. Transfections were performed using Lipofectamine 2000 according to the manufacturer's protocol. We added 0.8 μg of TOP-Flash or FOP-Flash plasmid to each well, and the ratio of pRL-sv40 to TOP-Flash or FOP-Flash was 50: 1. Forty-eight hours after transfection, the cells were washed twice with PBS and 200 μL of passive lysis buffer (PLB) (1: 4) added to each well. The cells were disassociated and concentrated in a table concentrator for 15 min at room temperature. The cell suspension was subsequently transferred to 1.5 mL EP tubes and centrifuged at 1,200 rpm at 4°C. During this time, the LAR and STOP solutions were prepared. Luciferase and Renilla values were measured using the Dul-Glo MAX^TM^ Luminometry System (Promega Corp., Madison, WI, USA). The relative ratio of TOP-Flash Firefly luciferase activity to pRL-TK Renilla luciferase activity was recorded as the strength of the transcriptional activity. The experiment was repeated three times and each group consisted of three replicates.

### MTT assays

After the transfected cells reached 80% confluence, they were washed twice with PBS, detached from the plates using 0.25% trypsin, and single cell suspensions collected. The cells were then counted and seeded in 96-well plates at a density of 3 × 10^3^ − 6 × 10^3^ cells/well (200 μL of the cell suspension/well, 6 parallel wells). We added 5 mg of the cell suspension to each well and cultured the cells for 4 h at 37°C. Following the incubation, the medium was aspirated, 150 μL of DMSO (Sigma-Aldrich) added to each well, and the plates gently agitated for 10 min. MTT reagent was then added at a concentration of 5 mg/mL in 20 μL (Sigma-Aldrich). The optical density (OD) values at 490 nm were measured using a spectrophotometer on days 1–6 and cell viability curves generated.

### Annexin V-FITC/propidium iodide (PI) staining

Forty-eight hours after transfection, the cells were digested with ethylenediamine tetraacetic acid (EDTA)-free trypsin, collected in flow cytometry tubes, and centrifuged at 1,000 rpm for 5 min. The supernatants were aspirated and the cells washed three times with cold PBS. The cells were then centrifuged once more and the supernatants discarded. We added 150 μL of Binding Buffer (Annexin-V-FITC Apoptosis Detection Kit, Sigma-Aldrich) and 5 μL of Annexin-V-FITC to each tube. The tubes were then mixed and incubated for 15 min at room temperature in the dark. Following the incubation, 100 μL of Binding Buffer and 5 μl of PI were added to each tube. Apoptotic cells were detected and analyzed by flow cytometry.

### Acridine orange staining

Transfected NSCLC cells were digested with trypsin and 0.3 mL of the cell suspension transferred to an EP tube. The cells were then incubated with 3 μL of acridine orange at a final concentration of 1 μM for 15 min at 37°C. Following the addition of 0.5 mL PBS, the tubes were centrifuged at 1,200 rpm for 5 min at 4°C. The supernatants were aspirated and the cell pellets resuspended in 1 mL PBS. After centrifuging the cell suspensions at 1,200 rpm for 5 min at 4°C, the supernatants were discarded and the cell pellets washed twice with 1 mL PBS. Following the final centrifugation, 10 μL of the solution at the bottom of each tube was retained and transferred onto a glass slide. The cytoplasm and nuclei of the cells exhibited uniform green fluorescence, DNA exhibited yellow-green fluorescence, and the RNA was dark red. Autophagic cells contained bright red cytoplasmic particles. Images were acquired on an inverted fluorescence microscope. Three high power fields were randomly selected in each group and the number of cells containing eosinophilic granules calculated.

### Quantitative real-time PCR (qRT-PCR)

The cells were cultured for 48 h after transfection. Total RNA was extracted from the cells in each group using E.Z.A.N. Fungal RNA miniprep kit according to the manufacturer's instructions (Ambion, USA). RNA was reverse transcribed into cDNA using high capacity RNA-to-cDNA kit (Applied Biosystems, Grand Island, NY, USA) according to the manufacturer's instructions (Fermentas, Iran). PCR was performed using Turboscript two-step quantitative RT-PCR kit and the manufacturer's protocol (Fermentas). Primers were synthesized by Invitrogen (Guangzhou, China) and the sequences are shown in Table 2. The qRT-PCR conditions were the following: initial denaturation at 50°C for 2 min, 95°C for 10 min, and 40 cycles of 95°C for 15 s, 56°C for 45 s. Relative gene expression was calculated using the 2^−ΔΔCt^ method, with the glyceraldehyde-3-phosphate dehydrogenase (GAPDH) as internal reference.

**Table 2:** Sequences of the qRT-PCR primers

Gene	Sequence
*β-catenin*	Upstream: 5′-GCTACTCAAGCTGATTTGATGGA-3′ Downstream: 5′-GGTAGTGGCACCAGAATGGATT-3′
*GSK-3β*	Upstream: 5′-AACACCAACAAGGGAGCAAA-3′ Downstream: 5′-GAGCGTGAGGAGGGATAAGG-3′
*LC3*	Upstream: 5′-GAGAAGCAGCTTCCTGTTCTGG-3′ Downstream: 5′-GTGTCCGTTCACCAACAGGAAG-3′
*Beclin1*	Upstream: 5′-AACCAGATGCGTTATGCCC-3′ Downstream: 5′-ATTGATTGTGCCAAACTGTCC-3′
*GAPDH*	Upstream: 5′-GGATTTGGTCGTATTGGG-3′ Downstream: 5′-GGAAGATGGTGATGGGATT-3′

qRT-PCR: quantitative real-time PCR; GSK-3β: glycogen synthase kinase-3β; LC3: light chain 3; GAPDH: glyceraldehyde-3-phosphate dehydrogenase.

### Western blotting

Forty-eight hours after transfection, the cells were washed three times with cold PBS, resuspended in protein extraction solution (100 μL/50 mL flask), and incubated on ice for 30 min. The lysates were centrifuged at 12,000 rpm for 10 min at 4°C and the supernatant collected in an 0.5 mL centrifuge tube and stored at −20°C. Total protein was quantified using a BCA kit (Pierce Biotechnology, Waltham, MA, USA). Proteins were stored at −70°C until use. SDS-PAGE was performed at 4°C for 1−2 h at 120V (resolving gel). Following electrophoresis, the separated proteins were transferred to PVDF membranes (Millipore, Billerica, MA, USA) at 4°C for 2 h. The membranes were blocked with 5% skim milk in tris-buffered saline tween (TBST) and incubated for 1−2 h at room temperature, followed by the addition of the primary antibodies: β-catenin (#9587, 1: 1000, Cell Signaling Technology, Beverly, MA, USA), p-β-catenin (ab27798, 1: 500, Abcam, Cambridge, UK), GSK-3β (ab93926, 1: 1000), p-GSK-3β^Ser9^ (ab131097, 1: 750), LC3 B (ab51520, 1: 3000), Beclin1 (ab207612, 1: 2000) and TUSC3 (ab77600, 1: 2000, Abcam), and incubated at 4°C overnight. After washing three times with TBST (10 min per wash), the membranes were incubated with a mouse secondary antibody (Abcam, Cambridge, UK) at room temperature for 1 h and then washed three times with TBST (10 min per wash). Finally, blots were developed using chemiluminescence and imaged on X-ray film.

### Immunofluorescence

One day before transfection, the cells were seeded in 6-well plates and stained once they reached 70% confluence. Cells were fixed with 2% paraformaldehyde for 10 min, washed three times with PBS (5 min per wash), permeabilized with 0.2% Triton X-100 (Sigma-Aldrich) for 10 min, and then washed three times with PBS (5 min per wash). After blocking the cells with 2% bovine serum albumin (BSA) for 30 min, the cells were washed twice with PBS (5 min per wash) and then incubated with a polyclonal anti-β-catenin primary antibody (ab209860, Abcam, Cambridge, UK) for 1 h at room temperature. The cells were washed three times with PBS (5 min per wash), and then incubated with the secondary antibody (Beijing Zhongshan Jinqiao Biotechnology Co., Ltd., Beijing, China) for 30 min at room temperature. After washing the cells four times with PBS (5 min per wash), the nuclei were stained with 0.5 μg/mL DAPI (Sigma-Aldrich) for 10 min. Finally, the cells were washed three times with PBS (5 min per wash). The coverslips were mounted using 20 μL of sealing agent and the cells imaged under a fluorescence microscope (× 200).

### Statistical analysis

Data were analyzed using SPSS version 18.0 (Chicago, IL, USA). Measurement data are expressed as the mean ± standard deviation (SD). Differences between multiple groups were analyzed by one-way analysis of variance (ANOVA), while pairwise comparisons were analyzed using least significant difference (LSD) *t*-tests. Enumeration data are presented as percentages or rates, and comparisons between groups were analyzed using chi-square tests. A *P* < 0.05 was considered statistically significant.

## References

[1] Kong L, Zhang P, Li W, Yang Y, Tian Y, Wang X, Chen S, Yang Y, Huang T, Zhao T, Tang L, Su B, Li F (2016). KDM1A promotes tumor cell invasion by silencing TIMP3 in non-small cell lung cancer cells. Oncotarget.

[2] Bai H, Mao L, Wang HS, Zhao J, Yang L, An TT, Wang X, Duan CJ, Wu NM, Guo ZQ, Liu YX, Liu HN, Wang YY (2009). Epidermal growth factor receptor mutations in plasma DNA samples predict tumor response in Chinese patients with stages IIIB to IV non-small-cell lung cancer. J Clin Oncol.

[3] Sequist LV, Martins RG, Spigel D, Grunberg SM, Spira A, Janne PA, Joshi VA, McCollum D, Evans TL, Muzikansky A, Kuhlmann GL, Han M, Goldberg JS (2008). First-line gefitinib in patients with advanced non-small-cell lung cancer harboring somatic EGFR mutations. J Clin Oncol.

[4] Cappuzzo F, Ligorio C, Toschi L, Rossi E, Trisolini R, Paioli D, Magrini E, Finocchiaro G, Bartolini S, Cancellieri A, Hirsch FR, Crino L, Varella-Garcia M (2007). EGFR and HER2 gene copy number and response to first-line chemotherapy in patients with advanced non-small cell lung cancer (NSCLC). J Thorac Oncol.

[5] Sun PH, Zhu LM, Qiao MM, Zhang YP, Jiang SH, Wu YL, Tu SP (2011). The XAF1 tumor suppressor induces autophagic cell death via upregulation of Beclin-1 and inhibition of Akt pathway. Cancer Lett.

[6] Fan X, Zhang X, Shen J, Zhao H, Yu X, Chen Y, Zhuang Z, Deng X, Feng H, Wang Y, Peng L (2016). Decreased TUSC3 promotes pancreatic cancer proliferation, invasion and metastasis. PLoS One.

[7] Horak P, Tomasich E, Vanhara P, Kratochvilova K, Anees M, Marhold M, Lemberger CE, Gerschpacher M, Horvat R, Sibilia M, Pils D, Krainer M (2014). TUSC3 loss alters the ER stress response and accelerates prostate cancer growth in vivo. Sci Rep.

[8] Ribeiro IP, Marques F, Caramelo F, Pereira J, Patricio M, Prazeres H, Ferrao J, Juliao MJ, Castelo-Branco M, de Melo JB, Baptista IP, Carreira IM (2014). Genetic gains and losses in oral squamous cell carcinoma: impact on clinical management. Cell Oncol (Dordr).

[9] Kratochvilova K, Horak P, Esner M, Soucek K, Pils D, Anees M, Tomasich E, Drafi F, Jurtikova V, Hampl A, Krainer M, Vanhara P (2015). Tumor suppressor candidate 3 (TUSC3) prevents the epithelial-to-mesenchymal transition and inhibits tumor growth by modulating the endoplasmic reticulum stress response in ovarian cancer cells. Int J Cancer.

[10] Chung KW, Kim SW, Kim SW (2012). Gene expression profiling of papillary thyroid carcinomas in Korean patients by oligonucleotide microarrays. J Korean Surg Soc.

[11] Yang L, Chen Y, Cui T, Knosel T, Zhang Q, Albring KF, Huber O, Petersen I (2012). Desmoplakin acts as a tumor suppressor by inhibition of the Wnt/beta-catenin signaling pathway in human lung cancer. Carcinogenesis.

[12] Li P, Zheng X, Shou K, Niu Y, Jian C, Zhao Y, Yi W, Hu X, Yu A (2016). The iron chelator Dp44mT suppresses osteosarcoma’s proliferation, invasion and migration: *in vitro* and *in vivo*. Am J Transl Res.

[13] Stinchcombe TE, Socinski MA (2009). Current treatments for advanced stage non-small cell lung cancer. Proc Am Thorac Soc.

[14] Pils D, Horak P, Gleiss A, Sax C, Fabjani G, Moebus VJ, Zielinski C, Reinthaller A, Zeillinger R, Krainer M (2005). Five genes from chromosomal band 8p22 are significantly down-regulated in ovarian carcinoma: N33 and EFA6R have a potential impact on overall survival. Cancer.

[15] Pils D, Horak P, Vanhara P, Anees M, Petz M, Alfanz A, Gugerell A, Wittinger M, Gleiss A, Auner V, Tong D, Zeillinger R, Braicu EI (2013). Methylation status of TUSC3 is a prognostic factor in ovarian cancer. Cancer.

[16] Kelleher DJ, Gilmore R (2006). An evolving view of the eukaryotic oligosaccharyltransferase. Glycobiology.

[17] Mohorko E, Glockshuber R, Aebi M (2011). Oligosaccharyltransferase: the central enzyme of N-linked protein glycosylation. J Inherit Metab Dis.

[18] Khalid AM, Asano A, Hosaka YZ, Takeuchi T, Yamano Y (2013). Tumor suppressor candidate TUSC3 expression during rat testis maturation. Biosci Biotechnol Biochem.

[19] Mohorko E, Owen RL, Malojcic G, Brozzo MS, Aebi M, Glockshuber R (2014). Structural basis of substrate specificity of human oligosaccharyl transferase subunit N33/Tusc3 and its role in regulating protein N-glycosylation. Structure.

[20] Ohtsubo K, Marth JD (2006). Glycosylation in cellular mechanisms of health and disease. Cell.

[21] Vanhara P, Horak P, Pils D, Anees M, Petz M, Gregor W, Zeillinger R, Krainer M (2013). Loss of the oligosaccharyl transferase subunit TUSC3 promotes proliferation and migration of ovarian cancer cells. Int J Oncol.

[22] Li YG, Liang NX, Qin YZ, Ma DJ, Huang CJ, Liu L, Li SQ (2016). Effects of RNAi-mediated TUSC3 silencing on radiation-induced autophagy and radiation sensitivity of human lung adenocarcinoma cell line A549 under hypoxic condition. Tumour Biol.

[23] Dihlmann S, von Knebel Doeberitz M. (2005). Wnt/beta-catenin-pathway as a molecular target for future anti-cancer therapeutics. Int J Cancer.

[24] Pinto D, Gregorieff A, Begthel H, Clevers H (2003). Canonical Wnt signals are essential for homeostasis of the intestinal epithelium. Genes Dev.

[25] Lee DK, Nathan Grantham R, Trachte AL, Mannion JD, Wilson CL (2006). Activation of the canonical Wnt/beta-catenin pathway enhances monocyte adhesion to endothelial cells. Biochem Biophys Res Commun.

[26] Zhu AJ, Watt FM (1999). beta-catenin signalling modulates proliferative potential of human epidermal keratinocytes independently of intercellular adhesion. Development.

[27] Muroyama Y, Kondoh H, Takada S (2004). Wnt proteins promote neuronal differentiation in neural stem cell culture. Biochem Biophys Res Commun.

[28] Ohno Y, Koyama H, Yoshikawa T, Takenaka D, Seki S, Yui M, Yamagata H, Aoyagi K, Matsumoto S, Sugimura K (2015). Three-way comparison of whole-body MR, coregistered whole-body FDG PET/MR, and integrated whole-body FDG PET/CT imaging: TNM and stage assessment capability for non-small cell lung cancer patients. Radiology.

[29] Scagliotti G, Kang JH, Smith D, Rosenberg R, Park K, Kim SW, Su WC, Boyd TE, Richards DA, Novello S, Hynes SM, Myrand SP, Lin J (2016). Phase II evaluation of LY2603618, a first-generation CHK1 inhibitor, in combination with pemetrexed in patients with advanced or metastatic non-small cell lung cancer. Invest New Drugs.

[30] Brown RS, Wahl RL (1993). Overexpression of Glut-1 glucose transporter in human breast cancer. An immunohistochemical study. Cancer.

[31] Chiou KR, Liu CP, Peng NJ, Huang WC, Hsiao SH, Huang YL, Chen KH, Wu MT (2008). Identification and viability assessment of infarcted myocardium with late enhancement multidetector computed tomography: comparison with thallium single photon emission computed tomography and echocardiography. Am Heart J.

